# Update Research Advances in the Application of Transcranial Magnetic Stimulation in the Treatment of Schizophrenia

**DOI:** 10.1155/2022/5415775

**Published:** 2022-09-12

**Authors:** Yanhai Wu, Zucheng Yang, Shu Cui

**Affiliations:** ^1^The Third People's Hospital of Fuyang, Fuyang 236000, China; ^2^Anhui Province Veterans Hospital, Bengbu 233000, China

## Abstract

Schizophrenia presents a chronic progressive course and requires long-term treatment. The current treatment of schizophrenia is mainly based on antipsychotic drugs, but drugs are ineffective for the negative symptoms and cognitive dysfunction of schizophrenia, and long-term medication may increase the burden on the endocrine and circulatory systems of patients. Repetitive transcranial magnetic stimulation is a noninvasive, painless, safe, efficacious, and economical physical therapy measure that has achieved good results in the treatment of schizophrenia. This paper reviews the progress of research on the clinical application of transcranial magnetic stimulation in the treatment of schizophrenia.

## 1. Introduction

Schizophrenia is a group of psychiatric disorders characterized by disorders of perception, thinking, emotion, volition, behavior, and other aspects and incoordination of mental activities, with a lifetime prevalence of about 1%. It can occur in people of any age but is most common in young adults [1], with 90% of cases starting between the ages of 15 and 55. The pathogenesis of schizophrenia is not yet fully understood, and it is widely believed that genetic factors, environmental factors, oxidative stress, body immunity, and neurobiochemical and structural brain abnormalities are involved. Cognitive abnormalities have also been found, as well as immune abnormalities, namely, increased levels of interleukin-induced C-reactive protein (CRP) [2, 3]. The course of schizophrenia is chronic and progressive, requiring long-term treatment. The main treatment is medication, but the side effects of long-term antipsychotic medication are high, resulting in low compliance with medication, increasing the burden on the endocrine and circulatory systems and other internal systems, and having limited effect on the negative and cognitive symptoms of schizophrenia, which affects the prognosis of patients [4] . Some patients with schizophrenia may also exhibit aggressive behavior that can harm themselves and threaten the safety of family members and health care workers [5]. Transcranial magnetic stimulation (TMS) uses electromagnetic induction technology to physically stimulate patients' neurological functions to improve clinical symptoms and promote cognitive function [6]. The present study reviews the progress of research on the application of transcranial magnetic stimulation in the treatment of schizophrenia to provide a clinical reference.

## 2. Transcranial Magnetic Stimulation

TMS is based on the principle of electromagnetic induction and electromagnetic conversion, in which the magnetic field generated by the electric current in the stimulation coil is applied to the central nervous system, resulting in induced currents in the cranial brain, thus causing changes in cerebral blood flow, brain metabolism, brain electricity, brain function, etc. This results in changes in cerebral blood flow, cerebral metabolism, EEG, and brain function. Repetitive TMS (rTMS) is one of the modalities of TMS. rTMS not only has a modulating effect on neurological functions during stimulation but also has a significant modulating effect after stimulation is stopped, and its effects on biochemical reactions, tissue structure, and physiological functions in the brain have a maintenance effect. rTMS is widely used in the treatment of psychoneurological diseases. It is widely used in depression, schizophrenia, and neurological disorders such as Alzheimer's disease because of its noninvasive, non-painful, and safe features [7]. Repetitive transcranial magnetic stimulation (rTMS) therapy is mainly used to excite or inhibit local cortical functions by changing the frequency of stimulation, respectively. High-frequency, high-intensity rTMS produces a sum of excitatory postsynaptic potentials, leading to abnormal excitation of nerves at the stimulation site; low-frequency stimulation has the opposite effect, treating the disease by regulating the balance between excitatory and inhibitory brain functions in both directions. The local nerves stimulated by rTMS have an impact on multi-site functions through the connection and interaction between neural networks; different intensity, frequency, stimulation site, and coil direction need to be adjusted to achieve good therapeutic effects for different patients' functional brain conditions.

## 3. The Need for TMS Technology in the Treatment of Schizophrenia

Clinical treatment of schizophrenia requires comprehensive treatment to control schizophrenic symptoms, reduce the impact of schizophrenia, delay disease progression, and improve the long-term quality of life of patients as the goal of treatment [8]. The clinical treatment of schizophrenia is based on antipsychotic medication, but because of the slow progression of schizophrenia and the lack of an effective cure, patients often have to take medication for a long time, so the side effects of the medication cannot be ignored [9]. The side effects of long-term anti-schizophrenia medication can cause insulin antagonism, adrenaline antagonism, cardiac arrhythmia, and other adverse reactions and can easily affect the balance of glucose and lipid metabolism, causing patients to have abnormal glucose and cholesterol metabolism indicators. As clinical research on schizophrenia treatment continues to unfold, TMS is widely used in the treatment of schizophrenia for its effectiveness, noninvasiveness, and high safety, and it has gradually become one of the preferred adjunctive modalities in the treatment of schizophrenia, which can effectively improve glucolipid metabolic indexes and serum neurotrophic factor levels and improve negative symptoms when combined with drugs [10].

## 4. TMS in the Treatment of Schizophrenia

### 4.1. Improvement of Negative-Positive Symptoms of Schizophrenia

The positive and negative symptom clusters of schizophrenia are the main target symptoms for clinical treatment, while the positive symptoms mainly include hallucinations, hallucinations, hallucinations, and delusions. High-frequency repetitive transcranial magnetic stimulation utilizes brief, potent magnetic field pulses in order to allow the magnetic field to rapidly traverse the skull, cortical folds, and adjacent cerebral white matter, promote neuronal excitation and the release of neurotransmitters such as dopamine, and improve local cortical metabolic abnormalities and regulate cortical activity, significantly improving patients' clinical symptoms. Su, Zongxia et al. [11] applied ziprasidone injection combined with repetitive transcranial magnetic stimulation (rTMS) to improve acute phase agitation symptoms in schizophrenia patients, and the positive and negative syndrome scale excitatory factor (PANSS-EC) scores at all time points 72 h after treatment were lower than those before treatment, which could effectively and safely improve acute phase agitation symptoms in schizophrenia patients, with some short-term efficacy continuation. Schizophrenia may also be related to structural abnormalities in the gray matter of the brain, which may be accompanied by a reduction in brain gray matter volume and density in the frontal and temporal lobes and other regions. Lin, Jing et al. [12] observed the effects on the efficacy and brain gray matter changes in patients with schizophrenia in the acute phase by paliperidone with high-frequency repetitive transcranial magnetic stimulation treatment for 8 weeks. This suggests that the use of paliperidone with high-frequency repetitive transcranial magnetic stimulation in the acute phase of schizophrenia can improve cerebral gray matter density and promote the recovery of cortical function, thereby alleviating clinical symptoms. The results of a previous study showed that 1HZ transcranial magnetic stimulation treatment resulted in improvements in phantom hearing and other neurocognitive performance in patients with schizophrenia, and that abnormalities in patients' global and local topological patterns were restored [13].

It is clear that research using rTMS to intervene in both positive and negative symptoms of schizophrenia leaves much to be desired, such as the fact that relevant studies are also small sample or open-label studies. Although the findings suggest that this is an emerging complementary treatment, the parameters and treatment sites are not uniform and further research is needed.

### 4.2. Improvement of Negative Symptoms of Schizophrenia

The negative symptoms of schizophrenia mainly manifest as emotional retardation, poor speech, lack of motivation, lack of anticipatory pleasure, and social withdrawal. The biological mechanisms of negative symptoms are complex, and there is a lack of effective targeted treatment. First-generation anti-schizophrenic drugs not only failed to improve negative symptoms but also aggravated negative symptoms, and second-generation anti-schizophrenic drugs could improve negative symptoms after they were widely used in the clinic, but the effect was not obvious. rTMS can affect the function of the stimulated local and functionally related distal compartment cortices to achieve regional reconstruction of cortical function, and the resulting biological effects can persist until some time after the cessation of stimulation, which has become a good tool for studying the functional reconstruction of neural networks and for exploring the treatment of negative symptoms in schizophrenia [14]. Most scholars now believe that low DA function in the left dorsolateral prefrontal cortex is associated with negative symptoms in patients. Mao, Jinyu [15] et al. used theta short burst rapid pulse (TBS) mode of repetitive transcranial magnetic stimulation (rTMS) for the treatment of negative symptoms in chronic schizophrenia, and the TBS mode, as a new stimulation mode of repetitive transcranial magnetic stimulation (rTMS) technique, was more consistent with neuronal firing patterns than the conventional mode and could reduce cortical hyperactivity more rapidly and possibly more effectively. The improvement of negative symptoms started at the end of 2 weeks after 4 weeks of treatment, suggesting that the improvement of psychiatric symptoms, especially negative symptoms, by rTMS in TBS mode contributes to the improvement of patients' social functions, thus enabling schizophrenic patients to better adapt to social life and return to society. Pu, Li et al. [10] applied high-frequency repetitive transcranial magnetic stimulation to treat schizophrenia patients with predominantly negative symptoms and the duration of its efficacy. After a 3-week period (15 sessions in total) of rTMS treatment at a frequency of 1 time/d and 5 times/week, schizophrenia patients with negative symptoms improved significantly, and the PANSS negative factor score was significantly lower at the end of the 11th week of treatment compared with that before treatment, and the curative effect of rTMS could maintain up to 2 months after treatment. Chang and colleagues conducted a randomized, double-blind, sham-controlled trial in stabilized schizophrenia patients to examine the efficacy of add-on hf-tRNS (2 mA; 100-640 Hz; 20 min) in improving negative symptoms. The result showed a significantly greater improvement in negative symptoms after active (17.11% reduction in PANSS-FSNS) than after sham stimulation (1.68% reduction in PANSS-FSNS), with a large effect size [16].

Studies using rTMS to intervene in negative symptoms of schizophrenia also suffer from the fact that parameters have not been standardized and there are fewer RCT-related studies; therefore, definitive efficacy cannot yet be derived and needs to be further explored.

### 4.3. Improvement of Depressive Symptoms in Patients with Schizophrenia

Most schizophrenia-associated depression is thought to be inherent in schizophrenia itself or secondary to antipsychotic medication or pessimism after schizophrenia has improved. Post-schizophrenic depression is defined as depressive symptoms that occur when schizophrenia has been diagnosed within the last year, when schizophrenia has improved but not recovered, and when depressive symptoms persist for more than 2 weeks, with an incidence of 20-70%. Some studies have reported that TMS has a high therapeutic safety in schizophrenia, and it may inhibit the re-uptake of 5-HT by the patient's central neurons through electromagnetic induction technology thus enhancing the patient's central neuronal dynamics, improving their stress resistance, and improving symptoms of depression, confusion, and anxiety [17–19]. The former applied transcranial magnetic stimulation at a frequency of 2 Hz to the left dorsolateral prefrontal lobe of the patient, based on the reference group, using a figure-of-eight coil with an MT value of 100%, and repeated 30 sequences at 5 s intervals, 5 times/week, 15 min/time, for a treatment period of 4 weeks; the latter applied with repeated transcranial magnetic stimulation using an “8” shaped coil with a stimulation frequency of 15 Hz at the left dorsolateral prefrontal lobe. 20 min per treatment, 5 times per week, 30 times in total. The efficacy of the treatment was significant. Chen, Qin [20] et al. applied high-frequency repetitive transcranial magnetic stimulation combined with escitalopram on male patients with post-schizophrenic depression and executive function, placing the center of the frontal “8” coil on the left dorsolateral prefrontal area (DLPFC) and tangent to the scalp, also using high-frequency stimulation at 10 Hz with a stimulation intensity of 90% MT, and the intervention was performed once a day for about 20 min, 5 times a week, and combined with pharmacological treatment for 4 weeks. The combination of high-frequency repetitive transcranial magnetic stimulation was shown to be more effective in reducing the depressive state and improving the executive function of the patients than single medication.

Studies have shown that rTMS has more definitive efficacy in treating depressive symptoms of schizophrenia. It is worth mentioning that rTMS has been approved by the US Food and Drug Administration (FDA) for the treatment of refractory depression and will have a good application in the field of treating depressive symptoms of schizophrenia.

### 4.4. Improvement of Cognitive Dysfunction in Schizophrenic Patients

More than [21] 85% of individuals with schizophrenia have severe and persistent cognitive impairment in speech, working memory, attention, and executive functioning. Cognitive dysfunction is one of the core symptoms of schizophrenia, and a significant correlation between the degree of cognitive dysfunction and the negative symptoms of schizophrenia has been clinically demonstrated. He, Shoubin [22] reported that patients with schizophrenia were stimulated with repetitive transcranial magnetic stimulation at a frequency of 20 Hz and the treatment site was the left dorsolateral prefrontal cortical region for 30 times, with a stimulation time of 5 s each time and an inter-stimulation interval of 30 s. The stimulation treatment time was controlled at 20 min, and the patients were stimulated once a day for 30 d. The improvement in cognitive function was assessed using the RBANS measure, which includes five dimensions, namely, visual breadth, verbal function, attention, delayed memory, and immediate memory, and effectively improved the cognitive function of patients with schizophrenia at the end of treatment. While Guan, Hengyong [23] et al. applied 10 Hz repetitive transcranial magnetic stimulation (rTMS) to treat clinical symptoms and cognitive function in demobilized veterans with chronic schizophrenia in a double-blind controlled study, 10 Hz rTMS did not show efficacy on clinical symptoms and cognitive dysfunction in chronic schizophrenia, probably the old age, long duration of illness, severe negative symptoms, especially severe social disconnection and lagging cultural level and structure are factors that influence the efficacy. Event-related brain potentials (ERPs) N400, P300, and mismatched negative waves (MMN) are effective in reflecting patients' cognitive function and have become a common research tool in cognitive science in recent years. Wang, Shaochang [24] et al. studied the effects of repetitive transcranial magnetic stimulation (rTMS) on event-related brain potentials (ERPs) N400, P300, and mismatched negative waves (MMN) in patients with schizophrenia, and patients were tested for ERPs before and after 25 sessions of rTMS treatment. The N400, MMN, and P300 wave amplitudes recovered after 25 rTMS treatments, and the patients' frontal areas showed a significant improvement in cognitive impairment. A study conducted by Thirthalli and colleagues noted that the additional use of MRI-guided rTMS provided no additional effect to the cognitive enhancement treatment; instead, the sham rTMS group showed greater cognitive improvement [25].

Currently, most of the relevant studies are also open-label trials, lacking high-quality randomized double-blind, controlled trials, and therefore, no clear conclusions on efficacy can yet be drawn, but it is still not a bad option for chronic schizophrenia with poor cognitive function.

## 5. Conclusion

rTMS is widely used in the treatment of psychiatric disorders, and stimulation of different areas may produce different effects. Stimulation of patients' temporoparietal areas may treat schizophrenic patients' hallucinatory symptoms, and stimulation of patients' frontal areas may improve patients' negative symptoms and cognition. In addition to the above treatment effects, some researchers have also explored the use of rTMS to intervene with wall skin symptoms in patients with schizophrenia, but because the relevant studies are very limited, they are not discussed in this article. These are all related to the functional activation of relevant brain regions and have been supported by neuroimaging, and the effect of transcranial magnetic stimulation on schizophrenia treatment can be confirmed. A number of other factors exist that may influence the efficacy of rTMS: combination medication, psychotherapy, and other therapies that may stimulate the brain. Although there are few controls applying pseudo-stimulation, there are differences in perception and the resulting psychological effects can influence the results and lead to errors. To date, there is a lack of high-quality RCTs of rTMS interventions in schizophrenia, and the influence of individual differences and placebo effects on the results cannot be excluded. Moreover, treatment parameters are not uniform and therefore no clear conclusions can yet be drawn about efficacy. Therefore, further confirmation of efficacy and further exploration of the optimal parameters of treatment are needed in large sample, multicenter RCT studies. In conclusion, the future prospect of rTMS application to psychiatric disorders is still worth looking forward to.
